RETRACTED

# Police violence and the health of black infants

**DOI:** 10.1126/sciadv.aax7894

**Published:** 2019-12-04

**Authors:** Joscha Legewie

**Affiliations:** Department of Sociology, Harvard University, Cambridge, MA 02138, USA. Email: jlegewie@fas.harvard.edu

## Abstract

Police use of force is a controversial issue, but the broader consequences and spillover effects are not well understood. This study examines the impact of in utero exposure to police killings of unarmed blacks in the residential environment on black infants’ health. Using a preregistered, quasi-experimental design and data from 3.9 million birth records in California from 2007 to 2016, the findings show that police killings of unarmed blacks substantially decrease the birth weight and gestational age of black infants residing nearby. There is no discernible effect on white and Hispanic infants or for police killings of armed blacks and other race victims, suggesting that the effect reflects stress and anxiety related to perceived injustice and discrimination. Police violence thus has spillover effects on the health of newborn infants that contribute to enduring black-white disparities in infant health and the intergenerational transmission of disadvantage at the earliest stages of life.

## Teaser

Analysis of 3.9 million birth records reveal spillover effects of police killings on the health of black infants.

## INTRODUCTION

On 9 August 2014, Officer Darren Wilson of the Ferguson Police Department fatally shot Michael Brown Jr., an 18-year-old African American man, in the city of Ferguson, Missouri, a suburb of St. Louis. The event and other well-publicized cases in 2014 brought renewed and national attention to police killings and police use of force more broadly. Recent data show that police kill about a thousand individuals each year in the United States and approximately 100,000 are admitted to hospital emergency rooms for nonfatal injuries inflicted by law enforcement officers (*1*, *2*). Police killings and other forms of police violence disproportionally affect minority groups and particularly black Americans (*1*, *3*, *4*). The rate of police killings is almost three times higher among blacks compared to whites (*3*). The consequences are stark for victims and their families, but the toll of police violence may extend to entire communities with spillover effects on those living nearby (*5*). This study examines the impact of in utero exposure to police killings of unarmed blacks in the residential environment on the health of black infants. To rule out alternative explanations and better understand the underlying sources of stress, it also compares the effects across racial/ethnic groups and examines the impact of police killings of armed and unarmed black, white, and Hispanic victims.

RETRACTED

Racial disparities in infant health are a major and persisting public health concern (*6*). The infant mortality rate is now twice as high among (non-Hispanic) black compared to white infants: 11.3 per 1000 black versus 4.9 per 1000 white babies (*7*, *8*). The rate of low birth weight (below 2500 g) for non-Hispanic black women is 1.96 times higher than that for white women with similar disparities in premature birth (<37 weeks gestational age) and other indicators of infant health (*9*). These racial disparities in infant health have long-term consequences for cognitive development, test scores, attention deficit hyperactivity disorder (ADHD), and other outcomes (*10*, *11*). A growing body of research highlights the importance of chronic stress related to experiences of racism and discrimination in explaining the persisting black-white disparities in infant health and ultimately individual outcomes throughout the life course (*12*–*18*).

Along these lines, police killings in the residential environment can trigger acute stress with negative consequences for infant health. Police killings evoke grief, collective anger, and hopelessness linked to perceived interpersonal discrimination in the form of unequal treatment by the police based on race and ethnicity. They are seen as a manifestation of structural racism or a broader system of laws, policies, and practices that maintain hierarchies and oppress racial minorities (*5*, *16*). The trauma, anxiety, hopelessness, and fear about future police encounters are all stressors. Accordingly, exposure to police killings in the residential environment or through news reports can trigger acute stress, which should be more pronounced for police killings of unarmed victims perceived as unjustified (*12*, *19*).

Recent research demonstrates some of these negative consequences of police killings and aggressive policing more broadly. For example, Bor *et al.* (*19*) show that police killings negatively affect mental health among black Americans. Related work documents the effect of police killings and aggressive forms of policing on educational outcomes, stress, and other health outcomes of black youth (*20*, *21*).

For black women who are pregnant, this exposure and related stress can shorten the length of gestation, affect birth weight, and increase the risk of other adverse health outcomes (*22*). The likely biological mechanism linking acute, environmental stressors during pregnancy, such as police violence in the residential environment, to birth outcomes is based on increased production of placental corticotrophin-releasing hormone (CRH) (*12*, *15*, *23*–*25*). Maternal and fetal stress triggers cells in the placenta and fetal membranes to produce CRH. CRH levels during gestation, in turn, are correlated with the risk of reduced gestational age at birth and low birth weight, presumably because CRH enhances prostaglandin production to promote childbirth (*23*, *24*). While previous research on the health consequences of stress largely focuses on chronic stress, acute stress during critical developmental stages such as the prenatal period might have similar consequences either because of similar biological responses or because acute stressors translate to chronic stressors (*10*). The negative effect of maternal stressors on birth outcomes likely depends on the distance to the event and the timing of exposure, with several studies suggesting that exposure to stressors in early pregnancy is particularly consequential (*26*–*28*).

RETRACTED

To examine the potential impact of police killings on infant health, this study presents a population-level analysis of vital statistics records from about 3.9 million births in California between 2007 and 2016. I link these birth records to incident-level data on 1891 police killings in California between 2005 and 2017 including 164 cases involving unarmed black victims (see fig. S1 for the geographic distribution of cases). The detailed geographic information on mothers’ residential location, together with the comprehensive dataset on police killings, makes it possible to study the effect of police killings during pregnancy in the residential environment on infant health. The analysis restricts the sample to singleton, in-state births to California residents and excludes cases with missing information on key variables. Restricting the sample to singleton births is important considering that twins and other multiples have lower birth weight and worse health at birth. Tables S1 to S3 show summary statistics for the sample of births. Materials and Methods includes further details on the data.

Estimating the effect of police killings on infant health is challenging because police killings are not random. They are linked to crime and other neighborhood characteristics, which might also affect birth outcomes. To overcome this challenge, this study relies on a preregistered, difference-in-difference (DD) approach with and without sibling comparison (*29*–*31*). The DD approach compares changes in birth outcomes for black infants in exposed areas born in different time periods before and after police killings of unarmed blacks to changes in birth outcomes for control cases in unaffected areas. The analysis distinguishes nine time periods for mothers who are exposed 18 to 13, 12 to 7, and 6 to 1 months before pregnancy; those who are exposed during the first, second, and third trimesters in utero; and those who are exposed 1 to 6, 7 to 12, and 13 to 18 months after birth. To safeguard the analysis against additional types of bias, this article uses a second estimation strategy based on mother fixed effects. This approach adjusts for all time-constant, observed, and unobserved maternal characteristics. It compares the infant health of siblings who were and were not exposed to police killings during pregnancy. To examine the role of spatial distance from police killings for the effect on infant health, this study defines exposure to police killings by 500-m intervals ranging from 1 to 6 km.

RETRACTED

The analysis focuses on two common measures of infant health. The first is birth weight measured in grams, and the second is gestational age measured in weeks based on the obstetric estimate of gestation. Birth weight and gestational age are related to infant mortality (*32*–*35*) and long-term outcomes such as cognitive development, test scores, ADHD, and others (*11*, *27*). In addition, the Supplementary Materials present results for high-risk infants and examine binary indicators for low birth weight (<2500 g) and preterm delivery (<37 completed weeks of gestation). Materials and Methods includes additional details about the statistical analysis, variables, and sample. Both estimation strategies and all outcomes were preregistered before data access. The preregistered analysis plan is available on the Center for Open Science Achieve at https://osf.io/x8by4 and a revision to the plan at https://osf.io/exzd5.

## RESULTS

Figure 1 shows the main findings for the effect of maternal exposure to police killings of unarmed blacks during pregnancy on the birth weight of black infants by trimester of exposure and distance to the incident. In utero exposure to police killings of unarmed blacks within 1 km of mother’s residence substantially reduces the birth weight of black infants by 50 to over 80 g, depending on the model specification and trimester of exposure. The size of this effect is substantial for exposure during the first and second trimesters. It corresponds to 0.10 to 0.15 standard deviations (sample standard deviation is 540.5 g) or a third to a fifth of the black-white gap in birth weight (sample gap is 242 g). The effect of exposure during the third trimester, however, is small and statistically insignificant, which is in line with previous research showing reduced effects of stressors at later stages of fetal development (*26*, *27*). The size of the effect is spatially limited and decreases with distance from the event. It is small and statistically insignificant in both model specifications at around 3 km. The negative effect during the first and second trimesters provides evidence that police killings of unarmed blacks significantly decrease the health of unborn black infants residing nearby. Figure S2 reports similar results for gestational age with a substantial negative effect of exposure during the first and second trimesters. However, the Supplementary Materials also report that the results for the binary outcomes of low birth weight and preterm birth are not as strong and partly statistically insignificant.

RETRACTED

**Fig. 1:** Effect of maternal exposure to police killings of unarmed blacks during pregnancy on the birth weight of black infants by trimester of exposure and distance to the incident. Symbols with lines represent point estimates with 95% confidence intervals from a DD model (left) and a DD model with sibling fixed-effects (right). The treatment indicator measures exposure to police killings by trimester of age. Additional covariates for exposure before and after pregnancy are omitted from the graphical presentation. Control variables include a linear county-specific trend, child’s gender, mother’s age and education, child parity, and fixed-effect terms for census tract, year-month, and mother ID for the sibling model. The number of cases is 246,018 for the DD model and 196,211 for the sibling model.

The causal interpretation of the DD results is based on the assumption that in the absence of police killings, birth outcomes would have been the same for exposed and unexposed infants. Several key findings support this assumption and a causal interpretation of the results. First, the trend in birth outcomes for infants exposed before and after pregnancy should be similar to infants in the control group who are never exposed. The models corroborate this common trend assumption with a series of terms that capture the difference in birth outcomes between the control and treatment group before and after pregnancy. Figure 2 presents the results. The findings demonstrate that there was no discernible difference in birth outcomes for infants exposed to police killings before or after pregnancy. The difference in birth weight is small for all and statistically insignificant for most of the estimates in both model specifications. However, birth weight is substantially lower for infants exposed to police killings of unarmed blacks during the first and second trimesters of gestation. Figure S2 reports similar results for gestational age. This temporal pattern is consistent with a causal interpretation of the results.

RETRACTED

**Fig. 2:** Effect of maternal exposure to police killings of unarmed blacks before, during, and after pregnancy on the birth weight of black infants. Symbols with lines represent point estimates with 95% confidence intervals from a DD model (left) and a DD model with sibling fixed-effects (right). See note for Fig. 1 about additional control variables. The number of cases is 246,018 for the DD model and 196,211 for the sibling model.

Second, the findings are stable across the DD model with and without a sibling fixed-effect term. The sibling model compares differences in birth outcomes for siblings who were and were not exposed to police killings. This additional specification reaffirms the findings based on different assumptions and safeguards the analyses against other types of bias.

Last, I rule out alternative explanations for underlying sources of stress by comparing the results across racial/ethnic groups and by examining the impact of police killings of armed blacks, and armed and unarmed white and Hispanic victims (*19*). Police killings of unarmed blacks can affect the health of black infants through two main channels: first, by creating stress and anxiety related to perceived injustice and discrimination or fear of future police encounters (*19*, *22*), and second, by provoking fear about general violence and crime as threats to personal safety (*26*). Suppose the effect of police killings of unarmed blacks is based on stress related to perceived discrimination. In this case, the effect should be more pronounced for police killings involving unarmed blacks and restricted to black infants (*19*, *22*). However, if the effect is largely driven by general violence and crime, then we would expect similar effects for other racial/ethnic groups independent of the victim’s race and potentially larger effects for police killings of armed victims, which signify serious criminal activity. Figure 3 presents the results for birth weight, and figs. S3 to S5 present the other outcome variables. The results show the effect of police killings of unarmed and armed black, white, and Hispanic victims on the birth weight of black, white, and Hispanic infants within 1.5 km of the incident. The findings indicate that the effect of police killings of unarmed Blacks is restricted to black infants. There is no discernible effect for police killings of armed blacks or unarmed and armed whites and Hispanics on any racial group. The effect sizes are mostly small, unrelated to the timing of exposure, inconsistent across the two model specifications and statistically insignificant for almost all of the estimated effects. This finding indicates that the effect is race specific and driven by perceptions of discrimination and structural racism instead of general threats of crime and violence. It rules out many alternative explanations such as violent crime or other confounders that operate similarly for police killings of unarmed and armed blacks.

RETRACTED

**Fig. 3:** Effect of maternal exposure to police killings of unarmed and armed blacks, whites, and Hispanics before, during, and after pregnancy on the birth weight of black, white, and Hispanic infants. Symbols with lines represent point estimates with 95% confidence intervals from a DD model and a DD model with mother fixed-effects. Confidence intervals for estimates with high uncertainty are cut off to limit the scale of the *y* axis. The number of cases for the DD model is 246,018 for black infants, 2,392,103 for Hispanic infants, and 1,297,071 for white infants. The number of cases for the DD model with a sibling fixed-effect term is 196,211 for black infants, 2,196,409 for Hispanic infants, and 1,241,755 for white infants. The full regression table is reported in tables S4 and S5.

The Supplementary Materials present a number of additional sensitivity analysis and robustness checks that were not specified in the preanalysis plan. These checks include different definitions of trimesters (table S7), redefining the time periods for exposure before and after pregnancy to cover 3 instead of 6 months (table S8) and addressing posttreatment selection bias related to residential mobility, miscarriage, and abortion (see Supplementary Text). The results confirm the main conclusions discussed here.

## DISCUSSION

The results provide causal evidence suggesting that extreme forms of police violence have broader consequences and spillover effects on the health of newborn infants. In utero exposure to police killings of unarmed blacks in the residential environment markedly reduced the health of black infants but not for other groups. Exposure to a single police killing of an unarmed black individual during pregnancy accounts for as much as a third of the black-white gap in birth weight. This finding indicates that police violence is an environmental stressor that contributes to the stark and enduring black-white disparities in infant health and therefore the intergenerational transmission of disadvantage at the earliest stages of life. Birth weight and gestational age are not only related to infant death in the short term (*32*–*35*); the consequences are long term with implications for cognitive development, test scores, ADHD, and others (*10*, *11*).

The findings have important implications for public policy. They highlight the broader implications and social costs of police use of fatal force far beyond the victim and their family members. Understanding the effects environmental stressors such as police violence have on infant health is important for the design and implementation of interventions that attempt to mitigate the negative consequences, reduce disparities in infant health and early child development, and promote a culture of health. In the past, public health initiatives to reduce disparities in infant health have centered on expanding access to prenatal care. The results and other recent research encourage policy makers and public health officials to broadly consider the stress, trauma, and anxiety experienced by racial/ethnic minorities such as the adverse consequences of police violence.

RETRACTED

The study also has important research implications. Racial inequality and discrimination are crucial reasons for adverse health outcomes and racial/ethnic disparities in health (*16*, *17*), but researchers largely rely on cross-sectional studies and struggle to identify the underlying processes that contribute to the observed relations (*16*). By estimating the effect of police killings on birth outcomes, this study highlights how the criminal justice system can adversely affect disparities in health. Linking vital records with incident-level event data showcases an innovative approach to study the health consequences of acute environmental stressors. This approach encourages future studies based on vital records, medical claims data, or other administrative health records to examine the impacts of an array of events on population health including the persisting black-white disparities in infant health.

## MATERIALS AND METHODS

This study relies on two data sources. The first are birth certificates for all births in California from 2007 to 2016 assembled by the Center for Health Statistics and Informatics at the California Department of Public Health. These birth records include every birth in California (about half a million per year) with information about birth weight and gestational age at birth as key measures of infant health, the date of birth, exact information on mothers’ residential location, and key maternal demographic characteristics such as race and ethnicity. For the geocoding of addresses on birth records, the ArcGIS Desktop geocoder was used. To identify full siblings in the sample, the study followed the procedure used by Liu *et al.* (*36*) based on California birth records from 1997 to 2007. This procedure exactly matches mother’s date of birth, father’s date of birth, and the first letter of the mother’s maiden name for all children born between 2007 and 2016. The analysis restricts the sample to singleton births considering that twins and other multiples have lower birth weight and worse health at birth. All analyses exclude cases with missing information on birth date, birth weight, gestational age, mother’s race, or mother’s residential address.

RETRACTED

The second data source is incident-level data on police killings in California between 2005 and 2017. These data rely on Fatal Encounters (*2*) and extensive additional coding. The coding procedure is described in the Supplementary Materials. The result of this procedure is a comprehensive database on officer-involved killings in California between 2005 and 2017. The database includes information on the date and geographic location of the incident, the race of the victim, and whether the victim was armed or unarmed.

Tables S1 to S3 present summary statistics for black, white, and Hispanic infants, respectively. The tables show summary statistics for all births and separately for infants exposed to police killings of unarmed and armed victims within 1, 2, and 3 km. Table S1 for black infants shows that infants exposed to police killings of armed or unarmed blacks have, on average, lower birth weight and a higher rate of premature births.

The analysis focuses on two common measures of infant health. The first is birth weight measured in grams, and the second is gestational age measured in weeks based on the obstetric estimate of gestation. Birth weight and gestational age are related to infant mortality (*32*–*35*) and long-term outcomes such as cognitive development, test scores, ADHD, and others (*11*, *27*). The measurement of birth weight is comparatively accurate, whereas gestational age is less reliable considering that it relies on the correct determination of the last menstrual period (LMP). The obstetric estimate of gestational age introduced by the National Centers for Health Statistics in 2003 and reported on California birth certificates starting in 2007 somewhat improves the measurement quality compared to previous estimates, although concerns persist (*37*). For this reason, the main text largely focuses on the findings for birth weight. The results for gestational age are reported in the Supplementary Materials, although the likely biological mechanism affects gestational age and preterm birth (*38*). In addition, the Supplementary Materials present results for high-risk infants and examine binary indicators for low birth weight (<2500 g) and preterm delivery (<37 completed weeks of gestation).

The goal of the analysis is to estimate the effect of maternal exposure to police killings of unarmed blacks on birth outcomes for black infants. Estimating the effect of police killings is challenging because police killings are not random. They are linked to crime and other neighborhood characteristics, which might also affect birth outcomes. To overcome this challenge, this study relies on a DD approach with and without sibling comparison (*29*–*31*, *39*). The estimation strategy and model specification are motivated by previous research on the effect of hydraulic fracturing on infant health (*31*) and the effect of police killings (*20*) and police surges (*21*) on student test scores.

RETRACTED

All models were estimated using a generalization of the within (fixed-effect) estimator for multiple high-dimensional categorical variables based on the lfe package in R (*40*). In particular, the models use the within transformation for the neighborhood and year-by-month fixed-effect term and for the mother fixed-effect term in the model with sibling comparison.

The DD approach leverages millions of birth records from California to compare changes in birth outcomes for black infants in exposed areas born in different time periods before and after police killings of blacks to changes in birth outcomes for control cases in unaffected areas. In particular, the models distinguish nine time periods for mothers exposed to a police killing 18 to 13, 12 to 7, and 6 to 1 months before pregnancy; those who are exposed during pregnancy by first, second, and third trimesters; and those who are exposed 1 to 6, 7 to 12, and 13 to 18 months after pregnancy. The regression models use clustered standard errors on the neighborhood level to address potential serial correlation problems (*41*). Formally, the models are specified as

$$y_{\text{icjt}}=\pi_{\mathrm{cj}}+\eta_{t}+\gamma_{c}\text{year}+\beta_{1}{\text{Near}}_{i}+\sum_{r=-3}^{5}\delta_{r}{\text{Exposure}}_{i,r}+\beta_{2}X_{\text{icjt}}+\varepsilon_{\text{icjt}}$$

where the dependent variables are birth outcomes for mother *i* in county *c* in census tract *j* and at year-by-month time period *t* (e.g., January 2014). The model includes a stable neighborhood effect π*_cj_* that controls for mean differences in birth outcomes across census tracts and a year-by-month time effect η*_t_* that captures differences in birth outcomes over years and months (e.g., January 2014) that are constant across all births such as seasonal fluctuations or general time trends. In addition, the model includes county-specific, linear time trends γ*_c_*year that captures different temporal trends in birth outcomes across California’s 58 counties. The vector ***X****_icjt_* consists of maternal and child characteristics. It includes sex of child coded as 0 for male and 1 for female, mother’s age (categorized as less than 20, 20 to 29, 30 to 34, or 35 years or older), mother’s education (categorized as less than high school, high school, some college, college, advanced degree, or missing), and child parity (first, second, third, fourth born or higher, parity missing).

RETRACTED

To estimate the effect of maternal exposure to police killings, the model includes two terms constructed separately for police killings of armed and unarmed blacks (*31*). The first is an indicator variable Near*_i_* that measures proximity of mother’s residence at time of birth to any police killing of unarmed blacks between 2005 and 2017 independent of the timing of the birth and the incident. It is coded as 1 if any police killing occurred within a specific distance *k* and 0 otherwise regardless of when the incident occurred. There is no a priori or theoretical way to derive the correct value of the distance parameter *k*. Instead, the spatial scale of a potential effect is an empirical question. Hence, the analysis defines exposure to police killings by increasing 500-m intervals ranging from 1 to 6 km. Note that the preregistered analysis plan includes distances as small as 0.25 km. This distance turned out to be infeasible because of the small number of births within this distance. Following the preanalysis plan, the Supplementary Materials nonetheless report the effect for 0.25 and 0.5 km in table S6. The Near*_i_* indicator measures whether at least one police killing occurred within the relevant distance.

The second is a set of nine indicator variables that measures the timing of maternal exposure to police killings of unarmed blacks within a specific distance *k*. The nine indicators distinguish between incidents that happened in different time periods before pregnancy, exposure during pregnancy by trimester of gestation (the key treatment indicators), and exposure during different time periods after pregnancy. All nine indicator variables are binary and coded as 1 if at least one police killing occurred during the specific time interval and within *k* kilometers of mother’s residence and 0 otherwise. Multiple of the nine indicator variables can be coded as 1 if multiple police killings occurred within *k* kilometers.

The three indicators for exposure before pregnancy are the time periods 18 to 13, 12 to 7, and 6 to 1 months before pregnancy. They are designated as *D_j_*, where *j* ranges from −3 to −1. While birth outcomes might be affected by exposure to police killings before pregnancy, infants are not exposed in utero.

The three treatment indicators measure exposure in utero by trimester of gestation within *k* kilometers of mother’s residence. They are defined as exposure during the first trimester *D*_0_, second trimester *D*_1_, and third trimester *D*_2_ of gestation. The three terms are the key treatment indicator and estimate the effect of maternal exposure to police killings by trimester of gestation. Trimesters are defined as consecutive 12-week intervals before the date of birth. This definition deviates from the medical definition based on the LMP. It ensures that the lengths of the third trimester and therefore the likelihood of exposure to police killings do not depend on gestational age, introducing a mechanical correlation between the treatment and outcome in the data (*42*). Table S7 shows the results from supplementary analyses exploring the sensitivity of the results to different definitions of trimesters. It includes an instrumental variable model using LMP-based trimesters for the three treatment indicators instrumented by exposure based on consecutive 12-week intervals used in the main analysis. Note that the preanalysis plan only refers to “trimesters” without specifying the coding of the time periods and without anticipating the problem related to the mechanical correlation between the treatment and outcome. The sensitivity analysis in table S7 ensures the robustness of the results to different definitions of trimesters.

RETRACTED

The final three terms are defined as exposed 1 to 6, 7 to 12, or 13 to 18 months after birth within *k* kilometers of the incident. The effect of the three indicators should be zero because the incident occurred after birth. The terms help us to evaluate the plausibility of the design. This specification makes it possible to examine changes in birth outcomes of black infants before and after police killings of unarmed blacks.

The second step of the analysis compares the estimates for maternal exposure to police killings of unarmed blacks with similar estimates for killings of armed blacks and unarmed and armed white and Hispanic victims on the health of black, white, and Hispanic infants. These analyses are based on separate exposure indicators for police killings involving black, white, and Hispanic victims and estimate the models separately for the sample of black, white, and Hispanic infants.

The second model specification uses a mother fixed-effect term to compare differences in birth outcomes for siblings who were and were not exposed to police killings. This additional specification reaffirms the findings based on different assumptions and safeguards our analyses against other types of bias. The sibling fixed-effect model restricts the sample to mothers with at least two births in the dataset. It is based on the following specification

$$y_{\text{icjt}}=\alpha_{i}+\pi_{\mathrm{cj}}+\eta_{t}+\gamma_{c}\text{year}+\beta_{1}{\text{Near}}_{i}+\sum_{r=-3}^{5}\delta_{r}{\text{Exposure}}_{i,r}+\beta_{2}X_{\text{icjt}}+\varepsilon_{\text{icjt}}$$

The mother fixed-effect term α*_i_* accounts for all observed and unobserved characteristics of the mother that are constant over time. As a consequence, the vector of covariates now only includes the child’s sex and excludes all characteristics that are constant or almost constant over time.

RETRACTED

The core assumption of both DD models is that, in the absence of police killings, changes in birth outcomes of exposed children would have been the same as changes in birth outcomes of children in control areas (common trend assumption). The estimates δ*_r_* for exposure before (*r* < 0) and after (*r* > 2) pregnancy make it possible to evaluate the common trend assumption indirectly. However, time-specific, neighborhood-level factors that are related to police killings and birth outcomes still threaten the identification strategy. Unobserved trends in crime rates or policing may account for both police shootings and changes in birth outcomes. From this perspective, a potential effect on birth outcomes is not caused by exposure to officer-involved killings but instead by changes in crime rates that increase police activity and officer-involved killings. While the model accounts for county-specific linear trends in birth outcomes and the specification of the exposure variable focuses on the 9 months of pregnancy, local crime waves (as opposed to general trends) that coincide with police killings are a potential threat to the identification strategy particularly because previous research links crime with birth outcomes (*26*).

To address this concern, I compare the effect of maternal exposure to police killings of unarmed blacks to the same effect for exposure to police killings of armed blacks. This falsification test rules out alternative explanations related to crime and other confounders (*19*). For example, the alternative explanation of a potential effect based on crime as a confounder has opposite implications for the types of police killings that are particularly consequential. If police killings affect birth outcomes simply because they reflect larger patterns in crime or because they provoke fear about crime and violence in general, then the effect of police killings involving armed victims should be more pronounced and the effect should be similar across racial/ethnic groups. However, if the effect is based on stress related to perceived discrimination, then the effect should be more pronounced for police killings involving unarmed blacks and it should be restricted to black infants. The analysis exploits these contradicting implications to rule out crime and many other potential confounders as alternative explanations.

RETRACTED

## Supplementary Material

http://advances.sciencemag.org/cgi/content/full/5/12/eaax7894/DC1

Download PDF

Preregistered analysis plan

Replication code

Police violence and the health of black infants

## SUPPLEMENTARY MATERIALS

Supplementary material for this article is available at http://advances.sciencemag.org/cgi/content/full/5/12/eaax7894/DC1 Supplementary Text Table S1. Sample characteristics for black infants. Table S2. Sample characteristics for white infants. Table S3. Sample characteristics for Hispanic infants. Table S4. Results from 36 DD models. Table S5. Results from 36 DD models with sibling fixed-effect. Table S6. Effect of exposure to police killing of unarmed blacks on birth weight of black infants for distances below 1 km. Table S7. Sensitivity analysis for various definitions of trimester. Table S8. Sensitivity analysis for different definitions of exposure to police killings before and after birth. Table S9. Effect of exposure to police killing of unarmed blacks during pregnancy on residential mobility for black mothers. Table S10. 2SLS models for effect of police killings of unarmed blacks during pregnancy within 1 km on birth weight of black infants. Fig. S1. Police killings in California, 2005–2017. Fig. S2. Effect of maternal exposure to police killings of unarmed blacks before, during, and after pregnancy on the gestational age of black infants. Fig. S3. Effect of maternal exposure to police killings within 1.5 km on gestational age in weeks by race/ethnicity of infant and characteristic of police killing. Fig. S4. Effect of maternal exposure to police killings within 1.5 km on low birth weight in weeks by race/ethnicity of infant and characteristic of police killing. Fig. S5. Effect of maternal exposure to police killings within 1.5 km on premature birth by race/ethnicity of infant and characteristic of police killing. Fig. S6. DD model for the effect of police killing of unarmed blacks on the number of births to black mothers. Preregistered analysis plan Replication code References (*43*–*48*)
